# Exploring Early Physical Examination Diagnostic Biomarkers for Alzheimer's Disease Based on Least Absolute Shrinkage and Selection Operator

This article has been retracted.

**DOI:** 10.1155/2022/3039248

**Published:** 2022-08-18

**Authors:** Hua Lin, Shiting Tang, Ling Liang, Liechun Chen, Chun Zou, Donghua Zou

**Affiliations:** ^1^Health Management Center, The Second Affiliated Hospital of Guangxi Medical University, Nanning, Guangxi 530007, China; ^2^Department of Neurology, The Second Affiliated Hospital of Guangxi Medical University, Nanning, Guangxi 530007, China; ^3^Department of Basic Medicine, Guangxi Medical College, Nanning, Guangxi 530022, China

## Abstract

Neurodegenerative diseases such as Alzheimer's disease (AD) are an increasing public health challenge. There is an urgent need to shift the focus to accurate detection of clinical AD at the physical examination stage. The purpose of this study was to identify biomarkers for AD diagnosis. Differential expression analysis was performed on a dataset including prefrontal cortical samples and peripheral blood samples of AD to identify shared differentially expressed genes (DEGs) shared between the two datasets. In addition, a minimum absolute contraction and selection operator (LASSO) model based on shared-DEGs identified nine signature genes (MT1X, IGF1, DLEU7, TRIM36, PTPRC, WNK2, SPG20, C8orf59, and BRWD1) that accurately predict AD occurrence. Enrichment analysis showed that the signature gene was significantly associated with the AD-related p53 signaling pathway, T-cell receptor signaling pathway, HIF-1 signaling pathway, AMPK signaling pathway, and FoxO signaling pathway. Thus, our results identify not only biomarkers for diagnosing AD but also potentially specific pathways. The AD biomarkers proposed in this study could serve as indicators for prevention and diagnosis during physical examination.

## 1. Introduction

Neurodegenerative diseases such as Alzheimer's disease (AD) are the leading cause of dementia, and AD-related dementia manifests as cognitive decline, accounting for more than 65% of all dementia cases [1, 2]. With the rapid aging of the global population, AD has become the focus of attention. According to world population statistics, in 2018, the elderly population in the world will reach 8.5%, and by 2050, this number will double. The main clinical manifestations of AD are inattention, memory loss, and the gradual decline of certain cognitive abilities, eventually resulting in self-reliance and death [3]. So far, there is no effective AD treatment method. AD can only treat the symptoms but not the root cause and delay of the development of the disease, which cannot prevent or reverse the disease [4, 5]. The development of AD has become a serious social problem, and its severity will affect the lives of patients and their families [6].

The differential diagnosis of AD is challenging [7, 8]. It is difficult to diagnose and monitor AD based on clinical data alone. At present, in AD diagnosis, biomarkers have become an important indicator of AD diagnosis [9–11]. The current detection methods used in AD pathology include positron emission tomography (PET) and cerebrospinal fluid (CSF) biomarkers of cerebrospinal fluid biomarkers [12, 13]. The widespread use of CSF- and PET-based imaging biomarkers remains limited due to the perceived invasive nature of lumbar puncture and the high cost and low availability of PET imaging [12, 14]. Therefore, there are a lot of research work on clinical markers and biomarkers combination, and now, we are working on noninvasive biomarkers. A large number of biomarkers play important roles in the transcriptional and posttranscriptional regulation of AD [15, 16]. Many studies are investigating the changes in brain mRNA levels in late AD [17]. However, there is a greater need for biomarkers that can diagnose disease at the time of early physical examination of AD.

In this study, we analyzed prefrontal cortical samples and peripheral blood samples from AD patients based on publicly available data to identify potential biomarkers of AD. LASSO models for nine genes (MT1X, IGF1, DLEU7, TRIM36, PTPRC, WNK2, SPG20, C8orf59, and BRWD1) with nonzero regression coefficients were constructed by identifying shared DEGs in prefrontal cortical samples and peripheral blood samples from AD patients. These signature genes can be used as biomarkers for early diagnosis of AD and provide the basis for disease progression monitoring, early physical examination, and early disease treatment.

## 2. Materials and Methods

### 2.1. Data Collection and Processing

AD-related datasets were downloaded from the Gene Expression Omnibus database (GEO, https://www.ncbi.nlm.nih.gov/geo/) [18]. The GSE33000 dataset [19] based on the GPL4372 platform included postmortem prefrontal cortex samples from a total of 310 AD patients and 157 normal subjects. In addition, the GSE97760 dataset [20] based on the GPL16699 platform includes peripheral blood samples from 9 AD patients and 10 matched healthy controls. GSE33000 and GSE97760 were used as the training set for this study. In addition, the GSE18309 dataset based on the GPL570 platform includes peripheral blood samples from 3 AD patients and 3 healthy controls. GSE18309 was used as the validation set for this study. Except for AD, all other samples were excluded. “Normalize between arrays” [21] was used in the limma package to normalize gene expression profiles. When multiple probes detect a gene at the same time, the expression value of each probe is obtained by the averaging method. The workflow of this paper is shown in Figure 1.

### 2.2. Differential Expression Analysis and Acquisition of Intersection Genes

In the GSE33000, GSE97760, and GSE18309 datasets, the differentially expressed genes (DEG) of AD patients and controls were analyzed using the limma package in *R* [21]. *P* < 0.01 was considered significant after adjustment for error discovery rate (FDR). DEGs from the intersection of the GSE33000 and GSE97760 datasets were identified as shared DEGs.

### 2.3. The Establishment of Least Absolute Shrinkage and Selection Operator (LASSO) and Receiver Operating Characteristic (ROC) Curves

LASSO has higher predictive value and less correlation; so, it can be used for optimal features of high-dimensional data [22, 23]. To study shared DEGs in postmortem prefrontal cortex and peripheral blood samples, we used the glmnet package (https://CRAN.R-project.org/package=glmnet) to extract expression profiles from shared DEGs to build a LASSO model. The expression values of the selected genes were weighted using the regressors of the LASSO analysis to create a model index for each sample using the following equation: index = ExpGene1∗Coef1 + ExpGene2∗Coef + ExpGene3∗Coef3 + ⋯ ^“^Coef^”^ is the regressor for the gene, derived from LASSO Cox regression, and “Exp” represents the expression of the gene. Next, the ROC was analyzed using pROC software to evaluate the AD recognition ability of the LASSO pattern [24]. In addition, to evaluate the diagnostic ability of the LASSO model feature genes, ROC curve analysis was performed in the training set using the pROC package, and expression analysis was performed using the *R* package ggplot2.

### 2.4. Enrichment Analysis

To explore the biological functions and pathways related to model signature genes, the Gene Ontology (GO) functions and Kyoto Encyclopedia of Genes and Genomes (KEGG) pathways were analyzed using the clusterProfiler package in *R* [25]. If *P* < 0.05, it can be regarded as significantly enriched.

### 2.5. Data Analysis and Statistics

All analyses in this study were performed using on the Bioinforcloud platform (http://www.bioinforcloud.org.cn). Differences were considered significant when the *P* value was less than 0.05.

## 3. Results

### 3.1. Identification of AD Prefrontal Cortex and Peripheral Blood Differentially Expressed Genes

In the GSE33000 dataset, a strong activation signal was shown in AD patients compared to healthy controls. The 2,096 DEG (50.3%) expression was significantly upregulated, and the 2,075 DEG (49.7%) expression was downregulated (Figures 2(a) and 2(c)). In addition, in the GSE97760 dataset, the 590 DEG (59.8%) expression was upregulated, and the 397 DEG (40.2%) expression was downregulated (Figures 2(b) and 2(d)). In the GSE33000 dataset and the GSE97760 dataset, a total of 33 intersecting genes were identified that may be shared DEGs by prefrontal cortical samples and peripheral blood in AD patients (Figure 2(e)). 33 DEGs shared by prefrontal cortical samples and peripheral blood in AD patients were visualized in the heat map (Figures 2(f) and 2(g)).

### 3.2. The LASSO Model Is a Potential Predictive Marker for AD

To establish the LASSO model, we extracted the expression profiles of 33 shared DEGs from the prefrontal cortex and peripheral blood of AD patients (Figures 3(a) and 3(b)). Using the LASSO method, a nonzero regression coefficient was found for 9 characteristic genes, with a value of lambda.min = 0.00126040395870055. The gene-based model index was created as the following equation: index = MT1X∗(−0.118329630586002) + IGF1∗4.47622713284553 + DLEU7∗0.579330259770386 + TRIM36∗2.16276722570743 + PTPRC∗(−0.604369904034408) + WNK2∗0.0412125079685932 + SPG20∗(−2.48528576171151) + C8orf59∗0.216147419776469 + BRWD1∗(−1.78870790466229). The area under the curve (AUC) of the model based on the 9 eigengenes was 0.937 in the GSE33000 training set (Figure 3(c)) and 1.000 in the GSE97760 training set (Figure 3(d)), indicating that the LASSO model can be used as a biomarker for AD. In addition, it was further confirmed in the validation set (GSE18309) with AUC = 0.667 (Figure 3(e)). This indicates that the genetic characteristics in the LASSO model have a certain relationship with AD and can be used as a biomarker for further detection.

### 3.3. Potential Biomarkers of AD for Prevention and Diagnosis

ROC curve analysis and expression profiles of nine signature genes from the training sets (GSE33000 and GSE97760) were further performed to explore the diagnostic efficacy of signature genes for AD (Figures 4(a) and 4(b)). These results validated the potential of these signature genes to diagnose AD.

### 3.4. Validation of the Biological Processes and Critical Pathways of AD

Further validation of the nine signature genes obtained from the LASSO model showed that DLEU7, IGF1, TRIM36, BRWD1, PTPRC, MT1X, and WNK2 were the most important hub genes (Figure 5(a)). These genes were enriched in biological processes such as regulation of neuroinflammatory responses and phagocytosis, such as the regulation of neuroinflammatory responses, positive regulation of the ERK1 and ERK2 cascades, the Fc-gamma receptor signaling pathway involved in phagocytosis, and biological processes regulating protein tyrosine phosphatase activity (Figure 5(b)). KEGG enrichment analysis revealed that these signature genes are involved in long-term depression, p53 signaling pathway, longevity regulatory pathway-multispecies, T cell receptor signaling pathway, HIF-1 signaling pathway, AMPK signaling pathway, and FoxO signaling pathway (Figure 5(c)).

## 4. Discussion

At present, there is no drug that can delay or inhibit the progression of AD, and no peripheral biomarkers have been found to detect the cause of AD early [26]. AD is a multigene, multipathway interacting disease whose etiology is still unclear. Furthermore, research on AD is very limited due to the inaccessibility of brain tissue from AD patients. Therefore, the analysis of the patient's brain tissue and peripheral blood is helpful for clinical research on AD. Currently, there is a clearer clinical understanding of the diagnosis of AD, and this therapy is expected to alleviate the progressive cognitive decline associated with AD [27]. At the same time, the application of bioinformatics technology to analyze various diseases provides a new method for clinical diagnosis and treatment. In this study, an open and open data platform was used to detect DEGs in postmortem prefrontal cortex and peripheral blood samples from AD patients and healthy controls and the regression coefficients of 0 without the LASSO model (MT1X, IGF1, DLEU7, TRIM36, PTPRC, WNK2, SPG20, C8orf59, BRWD1). These genes play a role in the early diagnosis of AD.

Some of these genes have been reported in AD. Insulin-like growth factor-1 (IGF1) promotes regeneration of neurons in the central nervous system (CNS) and peripheral nervous system (PNS) [28]. IGF1 is involved in the normal physiology of the body and the occurrence of diseases, especially the risk of dementia in AD patients is related to lower serum IGF1 levels. The higher the level, the more protection against neurodegeneration [29]. The biological role of IGF1 is mediated through IGF1R, and previous studies have shown that the high IGF1R expression in AD brain tissue is associated with clinicopathology [30]. Quan et al. identified BRWD1 and its corresponding biological processes involved in the development of AD by constructing an AD protein interaction network [31]. PTPRC was identified as Parkinson's disease biomarker [32] and in lung adenocarcinoma, latent tuberculosis, and ovarian cancer, PTPRC served as a key hub gene and was highly associated with disease [33–35]. These results suggest that the constructed LASSO model could provide valuable clues for researchers to identify key AD-related diagnostic biomarkers. However, more studies are needed to explore the functions of these genes in AD.

We conducted in-depth discussions on the biological mechanisms and pathways of AD. The results of functional enrichment showed that the characteristic genes of LASSO were involved in biological mechanisms such as regulation of neuroinflammatory response, positive regulation of ERK1 and ERK2, Fc-*γ* receptor involved in phagocytosis, and regulation of protein tyrosine phosphatase activity. In addition, KEGG enrichment analysis found that these genes were associated with long-term depression, including p53 signaling pathway, longevity regulatory pathway multispecies, T cell receptor signaling pathway, HIF-1 signaling pathway, AMPK signaling pathway, and FoxO signaling pathway. Many pathways are associated with AD. For example, the impact of HIF-1 signaling on neurodegeneration has been demonstrated [36, 37]. HIF-1 is an important regulator of hypoxic response in neurodegenerative diseases [38], and there is a lot of positive evidence that HIF-1 activation can delay the progression of AD [36, 39]. p53 is known to cause neuronal loss in AD, and p53 signaling is associated with AD [40]. Increasing evidence from neurodegenerative diseases suggests that activation of adenylate-activated protein kinase (AMPK) may have a broad neuroprotective role [41], and that the AMPK signaling pathway is associated with disease progression in AD patients [42]. Activation of FOXO may act as a homeostatic regulator in the stress response to prevent aging-related, including AD disease onset [43]. The nine signature genes and the biological processes and pathways they are involved in, obtained by the LASSO model in our study, suggest that these genes can serve as biomarkers for AD diagnosis.

Previously, studies have identified molecular signatures of blood cell origin and potential therapeutic targets through a comprehensive analysis of AD-related datasets [44]. Some studies have also analyzed brain tissue samples from AD patients by bioinformatics to look for biomarkers of AD [45–47]. Another study was used a web-based approach to identify biomarkers and therapeutic agents for AD [48]. And this study of ours still has merits compared to others. We combined datasets from prefrontal cortex samples and peripheral blood samples to identify signature genes for the diagnosis of AD, which is more accurate compared to signature genes identified directly in separate brain tissue samples or peripheral blood samples. Furthermore, blood biomarkers for AD have seemed elusive for many years, but recent results suggest that they may become a reality [49]. The results of the new high-sensitivity analysis show that across different groups, the data are clearly similar, although not precisely analyzed. In the peripheral blood confirmation set, the diagnostic markers of AD were confirmed, which laid the foundation for further research. However, the current research still has many shortcomings, such as the identification of specific genes that have not been tested experimentally. The role of these markers in the diagnosis of AD remains to be further studied. The pathogenesis of AD is complex, and one pathway alone cannot explain the occurrence of AD. More experiments are needed to confirm the current findings. Therefore, the results of this study should be carefully explained.

## 5. Conclusions

Our study shows that bioinformatics analysis can reveal some important insights about potential biomarkers in AD, identified as MT1X, IGF1, DLEU7, TRIM36, PTPRC, WNK2, SPG20, C8orf59, and BRWD1, which are indicators during physical examinations for preventive and diagnostic purposes.

## Figures and Tables

**Figure 1:** Research flow of this work.

**Figure 2:** Identification of differentially expressed genes shared by AD prefrontal cortex and peripheral blood. (a, b) Principal component analysis (PCA) of the GSE33000 dataset and GSE97760 dataset. (c, d) Volcano plot of AD controls in the GSE33000 (c) and GSE97760 (d) dataset, red represents upregulated genes, blue represents downregulated genes, and gray represents genes with no significant differential expression. (e) Differentially expressed genes (DEGs) shared by the GSE97760 dataset and the GSE97760 dataset. (f) GSE33000 heat map of the 33 shared DEGs in the dataset. (g) Heat map of the 33 shared DEGs in the GSE97760 dataset.

**Figure 3:** Construction of Lasso diagnostic model. (a, b) LASSO model. (c) ROC curve analysis of the training set (GSE33000). (d) ROC curve analysis of the training set (GSE97760). (e) ROC curve analysis of the validation set (GSE18309).

**Figure 4:** Potential biomarkers of AD for prevention and diagnosis. (a) ROC analysis and expression profile analysis of the signature genes identified by the LASSO model in the training set (GSE33000), *P* < 0.05. (b) ROC analysis and expression profile analysis of the signature genes identified by the LASSO model in the training set (GSE97760), *P* < 0.05.

**Figure 5:** Biological functions and pathways in which AD biomarkers are significantly involved. (a) The most important hub genes in the LASSO model. (b) Biological processes in which potential biomarkers of AD were involved. (c) KEGG signaling pathway in which potential biomarkers of AD were involved.

## Data Availability

The datasets supporting the conclusions of this article (GSE33000, GSE97760, and GSE18309) are available in the Gene Expression Omnibus (http://www.ncbi.nlm.nih.gov/geo).
